The article "Inhibition of melanogenesis by Gaillardia aristata flower extract" was published in 2015. Journal: BMC Complement Altern Med.

# Inhibition of melanogenesis by *Gaillardia aristata* flower extract

**DOI:** 10.1186/s12906-015-0972-1

**Published:** 2015-12-24

**Authors:** Minkyung Kim, Seoungwoo Shin, Jung-A Lee, Deokhoon Park, Jongsung Lee, Eunsun Jung

**Affiliations:** Biospectrum Life Science Institute, Eines Platz 11th FL, 442-13 Sangdaewon Dong, Seoungnam City, Gyunggi Do 462-807 Republic of Korea; Department of Genetic Engineering, Sungkyunkwan University, 2066, Seobu-Ro, Jangan Gu, Suwon City, Gyunggi Do 164-19 Republic of Korea

**Keywords:** *Gaillardia aristata*, Melanogenesis, Melanin, Tyrosinase, Skin-lightening effect

## Abstract

**Background:**

The purpose of the study was to determine the anti-melanogenic and anti-oxidant properties of *Gaillardia aristata* flower extract (GAE).

**Methods:**

Melanogenesis inhibition by GAE was investigated in cultivated cells and in a human skin model. In cultivated cells, the melanogenesis regulatory effect of GAE was evaluated using melanin content, intracellular tyrosinase activity and anti-oxidant characteristics. In addition, the expression of melanogenesis-related proteins was determined by western blot assay and real-time PCR.

**Results:**

GAE reduced the amount of melanin in B16F10 and normal human epidermal melanocyte cells and suppressed intracellular tyrosinase activity in a dose-dependent pattern. Also, GAE significantly decreased the expression of melanogenesis-related proteins (microphthalmia associated transcription factor, tyrosinase, tyrosinase-related protein-1, and dopachrome tautomerase). Real-time PCR results revealed a down-regulation of the mRNAs of these proteins. GAE possessed anti-oxidant characteristics as free radical-scavenging capacity and reducing power. In the three-dimensional human skin model, GAE applied to hyperpigmented skin significantly increased the degree of skin lightening within 2 weeks of treatment. The safety of GAE on human skin was confirmed.

**Conclusions:**

These results indicate the potential of GAE for use in suppressing skin pigmentation. We proposed GAE as a new candidate of anti-melanogenic and antioxidant agents that could be used for cosmetic skin care products.

## Background

Melanin secreted by melanocytes is the major pigment of human skin color in the basal layer of the epidermis. Melanin is crucial in photo-protection of human skin from harmful ultraviolet (UV) sunlight damage [1]. However, various hyperpigmented skin disorders result from the overproduction and subsequent accumulation of melanin, such as freckles, age spots, melanoderma, and senile lentigo, can be a distressing problem [2]. In melanin biosynthesis, the copper containing tyrosinase (TYR) enzyme catalyzes the hydroxylation of L-tyrosine to L-3,4-dihydroxyphenylalanine (L-DOPA) and the oxidation of L-DOPA to *o*-dopaquinone [3]. Microphthalmia associated transcription factor (MITF), tyrosinase-related protein-1 (TRP-1), and DCT are also essential for the production of melanin [4].

The article "Inhibition of melanogenesis by Gaillardia aristata flower extract" was published in 2015. Journal: BMC Complement Altern Med.

Melanogenesis produces the reactive oxidants including hydrogen peroxide (H_2_O_2_) and reactive oxygen species (ROS), which create oxidative stress in melanocytes. Certain ROS scavengers and inhibitors of ROS generation inhibit UV-induced melanogenesis and antioxidants like reduced glutathione (GSH) and ascorbic derivatives are applied to treat various skin problems such as depigmentation of hyperpigmented spots [5, 6]. Hence, antioxidants and free radical scavengers also play an important role in protecting human skin from the harmful effects by UV radiation as hyperpigmentation [7]. Development of effective anti-melanogenic agents with antioxidative capacity is a promising strategy to prevent or improve skin against damage due to UV radiation.

Depigmenting agents, such as arbutin [8] and kojic acid, have been used instead of hydroquinone to help prevent skin darkening. However, these compounds have undesirable side effects and can be weakly active [9–11]. Thus, it is important to develop new depigmenting agents as inhibitors of melanin formation that are derive from natural sources, which will lessen the likelihood of unrelated cytotoxicity or other side effects [12, 13].

In a preliminary study, we screened many herbal extracts for new melanogenesis inhibitors. The ethanol extract of *Gaillardia aristata*, a native plant in the sunflower family with a widespread geographic range and a prized ornamental plant, displayed strong inhibition of melanogenesis in B16F10 and HEMa-DP cells. The plant has a history of use in treating wounds and fever by Plateau Indian tribes [14].

Melanogenesis inhibition by *G. aristata* ethanol extract (GAE) has not been previously reported. We were particularly interested in its potential cosmetic applications. This study aimed to determine the antioxidative characteristics and the inhibitory effect of GAE on melanogenesis in cultivated cells and a three-dimensional (3D)-human skin tissue model.

## Methods

### Chemicals and reagents

Kojic acid, arbutin, α-MSH, 3,4-dihydroxyphenilalanine (L-DOPA), tyrosine, 3-(4,5-dimethyl-2-thiazolyl)-2,5-diphenyltetrazolium bromide (MTT), diphenyl-1-picrylhydrazyl (DPPH), 2,2'-azino-bis(3-ethylbenzothiazoline-6-sulphonic acid (ABTS), and dimethyl sulfoxide (DMSO) were purchased from Sigma-Aldrich (St Louis, MO, U.S.A.). Antibodies against TYR, TRP-1, DCT and MITF were obtained from Santa Cruz Biotechnology (Santa Cruz, CA, U.S.A.). Recombinant human stem cell factor (SCF) was supplied by ProSpec-Tany (Rehovot, Israel).

The article "Inhibition of melanogenesis by Gaillardia aristata flower extract" was published in 2015. Journal: BMC Complement Altern Med.

### Preparation of GAE

*G. aristata* flower seeds were perchased from wonyejongmyo (Korea) and we cultivated it in Jeju Island, Korea. After harvesting from July to August, the powdered *Gaillardia aristata* flower (28.9 g) was extracted overnight with 5 L of 70 % ethanol at room temperature and the supernatant was collected by filtration. Ethanol was removed by rotary vacuum evaporation (EYELA, Tokyo, Japan) and the extract (8.4 g) was lyophilized.

### DPPH scavenging activity assay

The antioxidant activity of GAE was first determined by measuring the DPPH scavenging ability [15]. The extract at various concentrations (25, 50, 100, 250, 500, and 1000 μg/mL) was added to 200 μL of DPPH (100 μM) solution. DPPH reaction with an antioxidant capable of hydrogen ion donation reduces DPPH. The resulting decrease in absorbance at 540 nm was recorded using a Gen 5™ UV-Vis spectrophotometer (BioTek, Winooski, VT, U.S.A.).

### ABTS^+^ scavenging capacity assay

The ABTS decolorization assay was done as previously described [16]. The assay relies on the generation of ABTS^+^ chromophore by oxidation of ABTS with potassium persulfate. The ABTS radical cation (ABTS^+^) was produced by reacting 7 mM stock solution of ABTS with 2.45 mM potassium persulfate and allowing the mixture to stand in the dark for at least 6 h before use. Absorbance at 734 nm was measured 30 min after the mixing of various concentrations of GAE (25, 50, 100, 250, 500, 1000 μg/mL) with 1 mL of ABTS^+^ solution.

### Determination of reducing capacity

The reducing power of the extract was determined as previously described [17]. The FRAP reagent was produced by mixing 300 mM acetate buffer (pH 3.6), 10 mM TPTZ solution, and 20 mM FeCl_3_⋅6H_2_O in a 10 : 1 : 1 ration and was prepared freshly at 37 °C. Different concentrations of GAE (25, 50, 100, 250, 500, and 1000 μg/mL) were individually mixed with FRAP reagent. The mixture was incubated at room temperature for 30 min in dark. The absorbance was measured at 595 nm in the UV-Vis spectrophotometer. Higher absorbance of the reaction mixture indicated greater reducing power.

### Determination of total phenolic content

Total phenolics were determined by an established assay [18]. Gallic acid was used to plot a standard curve. Various concentrations of GAE (50, 100, and 200 μg/mL) or gallic acid (50 and 100 μg/mL) dissolved in alkaline copper reagent was mixed with copper sulfate reagent, sodium dodecyl sulfate (SDS) solution, and sodium hydroxide solution in a 1:2:1 ratio, and incubated at room temperature. After 10 min, 0.5 mL of diluted Folin-Ciocalteu phenol reagent was added and then incubated for 30 min at room temperature. The absorbance of samples was measured 750 nm.

The article "Inhibition of melanogenesis by Gaillardia aristata flower extract" was published in 2015. Journal: BMC Complement Altern Med.

### Cell culture

B16F10 melanoma cells were cultured in Dulbecco's Modified Eagle's Medium (DMEM; Hyclone, Logan, UT, U.S.A.) with 10 % fetal bovine serum and penicillin/streptomycin (100 IU/50 μg/mL) in a humidified atmosphere containing 5 % CO_2_ in air at 37 °C. Primary cultures of normal human epidermal melanocytes (HEMa-DP; Cascade Biologics, Portland, OR, U.S.A.) derived from neonatal foreskin were cultured in Medium-254 (Cascade Biologics) supplemented with human melanocyte growth supplement (HMGS; Cascade Biologics) in a humidified atmosphere containing 5 % CO_2_ and 95 % air at 37 °C.

### Cell viability assay

Cell viability was determined by an established MTT-based assay. B16F10 melanoma cells and HEMa-DP cells were incubated with GAE for 5 days. Following treatment with MTT solution (1 mg/mL in phosphate buffered saline, PBS), the cells were incubated at 37 °C for 2 h. DMSO was added after the media was discarded and the absorbance was measured at 570 nm using the aforementioned a spectrophotometer.

### Determination of melanin content

B16F10 cells were first treated with GAE (10 and 20 μg/mL) in DMEM medium for 2 h followed by alpha-melanocyte-stimulating hormone (α–MSH; 50 nM) for an additional 72 h. HEMa-DP cells were incubated with GAE for 96 h. The cells were washed with PBS and lysed with 1 N NaOH for 1 h at 60 °C. Melanin content was estimated by the absorbance at 450 nm. Results were confirmed by three independent experiments. Before measuring the melanin content, cells were observed using a model TS-100 phase contract microscope (Nikon, Tokyo, Japan) and photographed using an attached TCH-5.0ICE digital camera (TUCSEN, Fujian, China) supported by ScopePhoto softeware (TUCSEN).

### Measurement of cellular tyrosinase activity

B16F10 cells were seeded at a density of 5 × 10^4^ cells per well in 6-well culture plates and incubated for 24 h. They were first treated with GAE for 2 h and then stimulated with 50 nM α-MSH for an additional 72 h. HEMa-DP cells were treated with GAE (10 and 20 μg/mL) and incubated for 5 days. The treated cells were washed twice using PBS and lysed with lysis buffer. Cell lysates were clarified by centrifugation at 5,000 rpm for 15 min at 4 °C. Enzyme activity was normalized to protein concentration, as determined by the Bradford assay. The cellular Tyrosinase and L-DOPA solution (0.1 M in sodium phosphate buffer) reaction were performed at 37 °C for 1 h. The absorbance at 450 nm was measured using the aforementioned spectrophotometer to monitor the production of dopachrome, corrected for auto-oxidation of L-DOPA.

The article "Inhibition of melanogenesis by Gaillardia aristata flower extract" was published in 2015. Journal: BMC Complement Altern Med.

### Tyrosinase zymography

Cultured cells were washed three times with PBS and harvested with lysis buffer (0.1 M sodium phosphate buffer (pH 6.8), 0.1 % Triton X-100, 1 % protease inhibitor cocktail). Protein content was determined with a Bradford assay using bovine serum albumin (BSA) as the standard. Equal amounts (20 μg) were mixed with sampling buffer and resolved by 10 % SDS-polyacrylamide gel electrophoresis. After electrophoresis, the gel containing tyrosinase activity was incubated with 0.1 M sodium phosphate buffer (NaH_2_PO_4_, pH 6.8) for 30 min at room temperature. The gel was incubated in the dark at 37 °C for 1 h after stained to 5 mM L-DOPA in 0.1 M sodium phosphate buffer.

### Tyrosinase luciferase reporter assay

To assay for tyrosinase promoter activity, B16F10 melanoma cells and HEMa-DP cells were transfected with tyrosinase reporter along with Renilla luciferase expression vector driven by the thymidine kinase promoter (Promega, Madison, WI, U.S.A.) using Superfect™ reagent (Qiagen, Valencia, CA, U.S.A.). After incubation for 24 h, cells were treated for 24 h with GAE. The cells were harvested and lysed, and the supernatants were assayed for luciferase activity using a Dual Luciferase Assay System (Promega, Madison, WI, U.S.A.).

### Western blotting

To measure melanogenesis pathways, 40 μg total protein was subjected to electrophoresis on a 10 % Bis-Tris gel (Invitrogen, Carlsbad, CA, U.S.A.). The resolved proteins were transferred to a nitrocellulose membrane that was blocked with 5 % BSA or 5 % skimmed milk in PBST (0.1 % Tween 20 in PBS) for 1 h. The membrane was incubated with the select primary antibody followed by incubation with the appropriate secondary antibody. Proteins were visualized using PowerOpti-ECL Western blotting Detection reagent (Anigen, Hwaseong, Korea). Protein bands were quantified with Image J software. β-actin were used as an internal control.

### Quantitative real-time PCR analysis

Total RNA samples were extracted using a RNeasy Midi kit (Qiagen) and aliquot (2 μg) of total RNA was reversed transcribed using a PrimeScriptII 1st strand cDNA Synthesis kit (Takara Bio, Shiga, Japan) according to the standard protocol. Quantitative PCR was performed with RT2 qPCR Primer Assay using the manufacturer’s protocol (Qiagen). Real-Time PCR was carried using SYBR green with the PCR Thermal Cycler MP device (Takara Bio). Each reaction was performed in triplicate. All human qRT-PCR primers were pre-designed, validated RT2 qPCR primer pairs (Qiagen) as follows. For human genes, TYR (PPH01771F), TRP-1 (PPH01770F), dopachrome tautomerase (DCT, PPH16498A), MITF (LPH40195A) and GAPDH (PPH00150F) were used. Relative gene expression was normalized to glyceraldehyde-3-phosphate dehydrogenase (GAPDH) mRNA and calculated with the ΔΔCT method.

The article "Inhibition of melanogenesis by Gaillardia aristata flower extract" was published in 2015. Journal: BMC Complement Altern Med.

### Histochemistry of reconstructed epidermis

A 3D-human skin tissue model (MatTek, Ashland, MA, U.S.A.) consisting of normal human-derived epidermal keratinocytes and normal human epidermal melanocytes was incubated in Long Life Maintenance medium (EPI-100-LLMM; MatTek, Ashland, MA, U.S.A.) containing GAE (100 and 200 μg/mL). The medium was replaced every 3 days for 14 days. Reconstructed human epidermis was fixed in 4 % paraformaldehyde using Fontana-Masson staining to stain melanin.

### Evaluation of inhibitory efficacy of GAE on the 3D-human skin model

The reconstructed human epidermis (MEL-300-B) was incubated with 20 nM SCF in the presence of GAE (100 and 200 μg/mL) for 14 days. Human recombinant SCF was added three times for 14 days. To measure the degree of pigmentation, L-values were measured using a CR-300 chromameter (Minolta, Tokyo, Japan).

### Human skin primary irritation test

The subject pool consisted of thirty healthy women and over ranging from 24 to 47 years of age. The subjects were required to satisfy all of the inclusion criteria and could not conflict with any of the exclusion criteria. Exclusion criteria were acute diseases, severe illnesses, pregnancy or lactation period, sensitization to ingredients of the test plaster, application of pharmaceutical products or skin care products with active ingredients until 4 weeks before testing, intake of drugs that possibly can interfere with skin reaction (steroids, anti-allegics, topical immuno-modulator, etc.) and extremely tanned skin. The subjects were required to be clearly informed regarding the nature of the study, the timetable, constraints and possible risks, both verbally and in writing. The average age of the subjects was 38.1 years. The subjects had no history of allergic contact dermatitis and had not used topical or systemic irritant preparations in the previous month. GAE (0.1 %) formulated with squalene was prepared and applied. The patches (chambers) stayed in place for 48 h. After patch removal, the condition of the skin at the patch sites were scored according to the terminology modified from Frosch & Kligman [19] and CTFA guidelines [20] as follows: 0 = no reaction; 1 = slight erythema, spotty of diffuse; 2 = moderate uniform erythema; 3 = intense erythema with ethema; 4 = intense erythema with edema and vesicles. Reactions are evaluated visually upon patch removal and at 30 min and 24 hours later. All assessments were performed under standard lighting conditions by a qualified research expert or dermatologist. This study was approved by the ethics committee of the DERMAPRO/Skin Research Center (Seoul, Republic of Korea).

The article "Inhibition of melanogenesis by Gaillardia aristata flower extract" was published in 2015. Journal: BMC Complement Altern Med.

### Statistical analysis

All data are expressed as mean ± SD. Differences between the control and treatment groups were evaluated by one-way ANOVA using SPSS software, version 22.0 (IBM Corporation, New York, NY, U.S.A.). A *p*-value < 0.01 was considered statistically significant.

## Results

### Antioxidant capacities of GAE

Four in vitro assays were performed to evaluate the antioxidant properties of GAE (Fig. 1). Radical-scavenging activity was assessed by the DPPH assay using vitamin C (50 μg/mL) and trolox (50 μg/mL) for comparative control. DPPH scavenging activity of the various concentrations of GAE (25-500 μg/mL) ranged from 25.39 ± 0.49 % to 96.55 ± 0.00 %, with an IC50 of 74.98 ± 0.48 μg/mL (Fig. 1a). The results indicated that free radical-scavenging activity of GAE in a dose-dependent manner. The ABTS^+^ scavenging capacity assay was performed to determine antioxidant activity. GAE at 200 μg/mL showed similar ABTS^+^ scavenging capacities as that of vitamin C (50 μg/mL) or trolox (50 μg/mL) (Fig. 1b). The IC50 of GAE was 110.79 ± 3.88 μg/mL. The results clearly indicated the antioxidant property of GAE. To measure the reducing activity of GAE, different concentrations of GAE (25-500 μg/mL) or trolox (50 μg/mL) were used. GAE at 500 μg/mL exhibited similar reducing capacity as trolox (Fig. 1c), indicating the reducing power of GAE. Total phenolic content of GAE was measured using gallic acid as the standard. The total phenolic content of GAE 200 μg/mL (103.38 ± 1.02 μg/mL) was higher than that of 100 μg/mL of gallic acid (96.21 ± 0.97 μg/mL) (Fig. 1d). This was probably due to some bioactive compounds, such as polyphenols including tannins and flavonoids, in GAE.

**Fig. 1:** The antioxidant properties of the effect of *Gaillardia aristata* flower extract (GAE). Radical scavenging activity was determined using different concentrations of GAE (25, 50, 100, 200, and 500 μg/mL) or vitamin C and trolox by DPPH (**a**) and ABTS^+^ (**b**). The effect of GAE was confirmed by measurement of reducing capacity (**c**) and total phenolic contents (**d**). Data are mean ± standard deviation. **p < 0.01 compared with the vehicle-treated group (*n* = 3)

### Effect of GAE on melanin production in HEMa-DP cells

The effect of GAE on human epidermal melanocytes proliferation was assessed using a MTT assay. Results are expressed as percent viability relative to control. The viability of human melanocytes treated with various concentrations of GAE compared to kojic acid is shown in Fig. 2a. No remarkable cytotoxicity was observed in human melanocytes treated with 5 and 10 μg/mL GAE. However, >20 μg/mL concentration was cytotoxic to human melanocytes. GAE at the nontoxic concentrations was used subsequently to determine the inhibition of melanogenesis in human melanocytes. We next performed human melanocytes were incubated with GAE at doses of 5-20 μg/mL for 96 h to investigate the effect GAE on melanin production. GAE produced a dose-dependent decrease in the melanin content of human melanocytes that exceeded the declines in kojic acid-treated samples (Fig. 2b).

The article "Inhibition of melanogenesis by Gaillardia aristata flower extract" was published in 2015. Journal: BMC Complement Altern Med.

**Fig. 2:** Cell viability (**a**) and melanin content (**b**) in human epidermal melanocytes incubated with the indicated concentration of GAE (5, 10, 20 μg/mL). Kojic acid are used as positive controls. Data are mean ± standard deviation. **p < 0.01 compared with the vehicle-treated group (*n* = 5)

### Effect of GAE on cellular tyroisnase inhibition in HEMa-DP cells

Cellular tyrosinase activity was determined to assess the depigmentig effect of GAE on human melanocytes because tyrosinase is crucial in melanogenesis. Kojic acid was used as a comparative control. The efficacy of tyrosinase inhibition by GAE (20 μg/mL) and kojic acid (60 μg/mL) was 25.62 ± 2.09 % and 19.21 ± 0.70 %, respectively (Fig. 3a). Additionally, the effects of GAE on cellular tyrosinase inhibition were determined by zymography. GAE treatment resulted in a dose-dependent reduction in the cellular tyrosinase (Fig. 3b). A luciferase reporter assay was carried out in human melanocytes to determine the antimelanogenesis activity of GAE. GAE inhibited tyrosinase luciferase reporter activation (Fig. 3c). These results indicated that GAE treatment significantly reduced cellular tyrosinase activity.

**Fig. 3:** Evaluations the effects of GAE on cellular tyrosinase activity by tyrosinase inhibition (**a**), zymography (**b**) and tyrosinase luciferase reporter assay (**c**) in Human melanocyte. Human melanocytes were treated with the indicated concentrations of GAE for 5 days and then the cellular tyrosinase activity was measured. The results are expressed relative to controls. Data are mean ± standard deviation. *p < 0.05 compared with the vehicle-treated group, **p < 0.01 compared with the vehicle-treated group (*n* = 3). Cell viability (**d**) and melanin content (**e**) were determined in B16F10 cells treated with GAE. Before measuring the melanin content, cells were observed using a contract microscope and photographed using an attached digital camera. Cellular tyrosinase activity was measured using tyrosinase inhibition (**g**), L-DOPA zymography analysis (**h**) and tyrosinase luciferase reporter assay (**i**). The results are expressed relative to controls. Data are mean ± standard deviation. ^##^ *p* < 0.01 compared with the vehicle-treated group, *p < 0.05 compared with the α-MSH-treated group, **p < 0.01compared with the α-MSH-treated group (*n* = 3)

The article "Inhibition of melanogenesis by Gaillardia aristata flower extract" was published in 2015. Journal: BMC Complement Altern Med.

### Evaluation of antimelanogenesis activity in B16F10

GAE exhibited antimelanogenesis in human epidermal melanocytes. B16F10 melanoma cells are widely-used to evaluate antimelanogenic effect of test materials because they are relatively easy to culture in vitro, and they share most of the melanogenic mechanisms of normal human melanocytes. To demonstrate the depigmenting activity of GAE in B16 melanoma cells, cell viability, melanin content, and tyrosinase activity were determined.

Cytotoxicity of GAE in B16F10 cells was measured using the MTT assay. When B16F10 cells were treated with 0-50 μg/mL GAE no significant cytotoxic effect was evident (Fig. 3d). Melanin levels and melanin pigmentation induced by α-MSH were reduced in a concentration-dependent manner by GAE treatment (Fig. 3e-f). To test whether GAE inhibited tyrosinase, a key enzyme catalyzing the rate-limiting step in melanin biosynthesis, tyrosinase zymography and tyrosinase luciferase reporter activation assays of enzyme activity were carried out in B16F10 melanoma cells. Tyrosinase activity in GAE-treated and cultured B16F10 melanoma cells was suppressed in a dose-dependent pattern (Fig. 3g-i).

### Effect of GAE on melanogenesis-related proteins and gene expression

To test whether GAE does regulate the expression of melanogenesis-related proteins, HEMa-DP cells were treated with GAE (10 and 20 μg/mL) for 5 days. TYR, TRP-1, DCT, and MITF levels were assayed by Western blot (Fig. 4a). Compared with untreated control cells, GAE treatment at 20 μg/mL significantly reduced TYR, TRP-1, DCT, and MITF level in a dose-dependent manner (Fig. 4b-e). Additionally, the effects of GAE on expression of melanogenic genes were tested using real-time PCR. mRNA levels of MITF and its downstream genes, TYR, TRP-1 and DCT, were reduced by GAE (Fig. 4f). GAE may contribute to the inhibition of melanogenesis by regulating the expression of tyrosinase-related genes as wells as MITF.

**Fig. 4:** Inhibitory effects of GAE on expression of melanogenesis-related protein and mRNA. **a** Western blot assay were performed to estimate protein expression levels of **b** tyrosinase (TYR), **c** tyrosinase-related protein-1 (TRP-1), **d** DCT, and **e** MITF. Protein loading amounts were confirmed by β-actin expression and **f** the mRNA levels were examined by real time RT-PCR using glyceraldehydes 3-phosphate dehydrogenase (GAPDH) as control. Data are mean ± standard deviation. **p < 0.01 compared with the vehicle-treated group (*n* = 3)

The article "Inhibition of melanogenesis by Gaillardia aristata flower extract" was published in 2015. Journal: BMC Complement Altern Med.

### Effect of GAE in human epidermal equivalents

To more closely approximate human usage, a reconstructed human skin model was used to investigate the depigmenting activity of GAE. Kojic acid was the positive standard, consistent with its common use for skin depigmentation therapy. As shown in Fig. 5, the level of melanin decreased significantly following GAE treatment. The depigmenting activity of 200 μg/mL GAE was comparable to that of 2 % kojic acid.

**Fig. 5:** GAE significantly decreases the level of melanin pigmentation in reconstructed epidermis. Reconstructed epidermis was exposed to GAE or kojic acid for 2 weeks and pigmentation was observed upon Fontana-Masson (FM) staining. Data are mean ± standard deviation. **p < 0.01 compared with the vehicle-treated group (*n* = 3)

### Effect of GAE on SCF-stimulated pigmentation in human epidermal equivalents

Hyperpigmentation causes skin darkness and medical disorders by melanocyte activity involved in UV damage or post-inflammation [21, 22]. Several cytokines and chemokines, such as SCF and endothelin-1 (ET-1), function in hyperpigmentary mechanism related to UVB exposure or senile lentigo [23, 24]. Therefore, we examined the inhibition of GAE on melanogenesis induced by SCF in normal human epidermal melanocytes. Human epidermal equivalents were treated with GAE (100 and 200 μg/mL) or SCF (20 nM) and skin lightening index was recorded. The color of the human epidermal equivalents treated with 200 μg/mL GAE was lighter than that of the untreated control. Furthermore, the addition of SCF gradually stimulated visible pigmentation over 14 days of treatment. During the SCF-induced stimulation of pigmentation, the addition of either concentration of GAE distinctly reduced the increase in visible pigmentation over 14 days (Fig. 6a-b).

**Fig. 6:** GAE-mediated inhibition of melanogenesis induced by SCF in normal human epidermal melanocytes. Reconstructed epidermis were cultured with GAE and SCF (20 nM) for 14 days. Images were exhibited using a microscope **a**. L-values of cell pigmentation were measured using a chromameter (CR-300, Minolta) **b**. Data are mean ± standard deviation. ^##^ *p* < 0.01 compared with the vehicle-treated group, **p < 0.01 compared with the SCF-treated group (*n* = 3)

### Human skin primary irritation test of GAE

Natural products including plant derived extracts and naturally derived substances may have side effects such as cutaneous irritation and allergic hypersensitivities. Skin primary irritation test in humans is the typical way of determining substance safety. To evaluate the irritation effect of GAE for clinical applications to human skin, a patch test was performed. The data of 31 subjects was collected and analyzed. As shown in Table 1, GAE did not show any skin reaction at 30 min and 24 h after patch removal in all subjects. This result indicated that GAE is safe to use as a potential alternative for cosmetic ingredient.

The article "Inhibition of melanogenesis by Gaillardia aristata flower extract" was published in 2015. Journal: BMC Complement Altern Med.

**Table 1:** Human skin primary irritation test

No.	Test Material	48 h					72 h					Reaction grade^b^		
		±	1+	2+	3+	4+	±	1+	2+	3+	4+	48 h	72 h	Mean
1	Squalene	-^a^	-	-	-	-	-	-	-	-	-	0	0	
2	GAE (0.1 %)	-	-	-	-	-	-	-	-	-	-	0	0	

^a^No reaction; ^b^Reaction grade = Σ [{Grade × No. of Responders}/{4(Maximum grade) × 30 (Total subject)}] × 100 × (1/2)

## Discussion

Although kojic acid and arbutin are common skin whitening products, there is a need to find safer and more effective skin lightening agents because of the carcinogenic possibility of kojic acid [9, 10] and weak photostability of arbutin [25]. In this study, GAE showed good antimelanogenic activity similar to those of chemicals, and no adverse skin reactions including erythema, burning, or pruritus. Based on these results, GAE can be used as alternative skin-lightening agent to kojic acid and arbutin.

It is necessary to confirm the effectiveness of the newly discovered anti-melanogenesis inhibitors in a 3D skin model. Histological change due to depigmenting effect of GAE was observed using Fontana-Masson staining in human epidermal equivalents. GAE inhibited melanin production more strongly than kojic aicd in human epidermal equivalents. In addition SCF-induced melanin production was decreased in the GAE-treated group.

Melanogenesis is regulated by keratinocyte-derived mediators such as α-MSH, basic fibroblastic growth factor, SCF, ET-1. Keratinocytes also produce cytokines, such as interleukin (IL-6) and tumor necrosis factor-α (TNF-α), which function as paracrine inhibitors in human melanocytes. The mechanism of epidermal hyper-pigmentation occurs by the increased expression level of ET-1 and SCF, or the decreased expression of TNF-α and IL-6. In particular, SCF and ET-1 are germane to the hyper-pigmentary mechanism by UVB-induced melanin synthesis [26–30]. Presently, GAE inhibited SCF-stimulated pigmentation in human epidermal equivalents. SCF stimulates MITF expression, which leads to up-regulate tyrosinase activity. GAE inhibited MITF expression and tyrosinase activity in melanocytes. Further studies will be required to elucidate the SCF pathway related to antimelanogenic activity of GAE.

In this study, GAE additionally exhibited an antioxidant effect and had reducing power. In addition, as the amount of total phenolics of GAE (200 μg/mL) was higher than that of gallic acid (100 μg/mL), the antioxidant capacity of GAE perhaps derived from polyphenolic constituents of GAE. Flavonoids including polyphenol have antioxidant and antimelanogenic activities [31–33]. The main mechanism of flavonoids having the depigmenting effect may be the ROS-scavenger properties and the ability to chelate metals at the active site of metalloenzymes [34].

The article "Inhibition of melanogenesis by Gaillardia aristata flower extract" was published in 2015. Journal: BMC Complement Altern Med.

## Conclusions

GAE potently inhibits melanin production by reducing TYR, TRP-1, DCT and MITF expression in melanocytes. This antimelanogenic effect was also confirmed in B16 melanoma cells and in a 3D skin model. In addition, GAE has the apparent antioxidant capacity and no skin primary irritation in humans. These findings imply that GAE can be developed as an anti-hyperpigmentation and antioxidant agent in human skin care products.
